# Design and Optimization of the Circulatory Cell-Driven Drug Delivery Platform

**DOI:** 10.1155/2021/8502021

**Published:** 2021-09-22

**Authors:** Pengyu Gao, Dan Zou, Ansha Zhao, Ping Yang

**Affiliations:** Key Laboratory for Advanced Technologies of Materials, Ministry of Education, School of Material Science and Engineering, Southwest Jiaotong University, Chengdu 610031, China

## Abstract

Achievement of high targeting efficiency for a drug delivery system remains a challenge of tumor diagnoses and nonsurgery therapies. Although nanoparticle-based drug delivery systems have made great progress in extending circulation time, improving durability, and controlling drug release, the targeting efficiency remains low. And the development is limited to reducing side effects since overall survival rates are mostly unchanged. Therefore, great efforts have been made to explore cell-driven drug delivery systems in the tumor area. Cells, particularly those in the blood circulatory system, meet most of the demands that the nanoparticle-based delivery systems do not. These cells possess extended circulation times and innate chemomigration ability and can activate an immune response that exerts therapeutic effects. However, new challenges have emerged, such as payloads, cell function change, cargo leakage, and in situ release. Generally, employing cells from the blood circulatory system as cargo carriers has achieved great benefits and paved the way for tumor diagnosis and therapy. This review specifically covers (a) the properties of red blood cells, monocytes, macrophages, neutrophils, natural killer cells, T lymphocytes, and mesenchymal stem cells; (b) the loading strategies to balance cargo amounts and cell function balance; (c) the cascade strategies to improve cell-driven targeting delivery efficiency; and (d) the features and applications of cell membranes, artificial cells, and extracellular vesicles in cancer treatment.

## 1. Introduction

According to the World Health Organization (WHO) report in 2018, cancer remains one of the top 10 global causes of death [1]. Because tumor cells lead to immortality, migration, and loss of contact inhibition, most patients only benefit from combined treatments, such as surgery, chemotherapy, radiotherapy, and immune therapy. In terms of prevention of the recurrence and metastasis of unresectable tumors, cancer treatment still faces many challenges, especially with respect to nonsurgery therapies and diagnoses. Currently, ensuring the delivery of sufficient cargos to lesions precisely and effectively is an important issue for nonsurgery therapies and diagnoses [2, 3].

Earlier, a nanoparticle-based drug delivery system (DDS) was developed, which improved the solubility of chemotherapeutics and lessened their toxicity to normal tissues. From intravenous injection to tumor sites, cargo-loaded nanoparticles (NPs) go through a CAPIR cascade: Circulation, Accumulation, Penetration, Internalization, and Drug Release [4]. In the blood circulatory system, naked NPs are vulnerable to the reticuloendothelial system (RES). Recently, they have also been found to be hitchhiked by circulating cells before being phagocytosed by RES tissues [5]. Modifying NPs with stealth molecules, such as polyethylene glycol (PEG) [6] and polyglycerol (PG) [7], has been reported to reduce the clearance risk and overcome some pharmacokinetic-related issues. During the accumulation and penetration to stages, it has been recognized that 10–1000 nm NPs can make full use of enhanced permeability and retention (EPR) effects via intercellular extravasation to accumulate at and penetrate tumor tissues [3]. When NPs are coupled with targeting molecules (e.g., Fe_3_O_4_, short peptides, and antibodies), then the passive delivery system can be transformed into an active system [3, 8]. However, a recent study revealed that approximately 97% of NPs themselves accumulate in an active transcellular manner through endothelial cells (ECs) [9], which advances our understanding of the NP accumulation mechanism in tumors to a new level. When NPs arrive at the lesion, their neutral surface charge, particle size below 100 nm, and nonspherical shape can further increase the penetration and internalization rates [10]. Additionally, NPs have made it possible to maintain the drug at a certain concentration in the tumor tissues, via self-diffusion, degradation, or a stimulus response, such as a response to pH, an enzyme, light, radiation, a magnetic field, or ultrasound [11]. Compared to free cargos, an NP-based DDS protects them from the phagocyte system; has an enhanced *in situ* cargo concentration, especially for hydrophobic systems; has facilitated specific delivery for one/multiple cargos; and has release control. The NP-based DDS has improved the evolution of nonsurgery therapies and diagnosis strategies.

NPs exhibit the substantial potential to deliver drugs, yet outstanding performance is limited to reducing side effects of anticancer drugs and not enhancing therapeutic efficacies [4]. The basic reason for this is that the NP-based DDS has long suffered from rapid clearance from the RES and a low targeting delivery efficiency of 1% [10]. Low targetability partially results from interstitial fluid pressure, which is 10–40 times higher in tumor cells than in normal cells [10], and from heterogeneous EPR, wherein the EPR mechanism has failed in tumors, such as lymphoma subtypes [12]. NPs smaller than 20 nm penetrate deeper, but this size is in a perfect clearance range for the RES [4]. The blood-brain barrier (BBB) is another obstacle for brain tumors because NPs scarcely cross it [13]. Furthermore, in the BBB, shear stress also impedes the distribution of NPs. NPs are taken up in a flow speed-dependent manner; i.e., the faster the flow, the lower the uptake. Various shear stresses in tumor vasculature may result in a heterogeneous NP distribution [14]. Because controlled release and biocompatibility are also required, an NP-based DDS faces a crucial challenge to be multifunctional [8] simultaneously.

In the past twenty years, the cell-driven DDS has gained much attention as an alternative approach. Additionally, an increasing number of studies have shown that a cell-driven DDS can address the major concerns of NP-based systems [15, 16]. Endogenous cells have a long circulation time with low toxicity risk and are not removed by the RES or kidneys [17]. Immune and stem cells can chemomigrate and transverse blood barriers, including the BBB; thus, they can penetrate the deep tumor matrix [18] instead of EPR-dependent intracellular extravasation [12]. These results have provided a new DDS and shed light on improving circulating and targeting delivery efficiency *in vivo* for cancer diagnosis and therapy. This article will focus on (a) the properties of circulatory cells, mainly red blood cells (RBCs), leukocytes, and mesenchymal stem cells (MSCs); (b) the loading strategies for balancing payload amounts and cell functions; (c) the cascade strategies for improving cell-driven targeting delivery efficiency; and (d) the cell membrane and small extracellular vesicles (EVs) as drug carriers for targeting delivery.

## 2. Utilizable Properties of Circulatory Cells

A tumor is a neotissue, which obtains nutrients and oxygen via RBC-involved angiogenesis. Tumors are also an inflammatory microenvironment, which is flooded with diverse cells, including MSCs [19] and different leukocytes (monocytes (MOs) [20], macrophages (MAs), neutrophils (NEs), natural killer cells (NKs), and T and B lymphocytes [21]). A large number of RBCs, leukocytes, and MSCs exist in the blood; it is a good source for drug delivery carriers, as listed in Table 1 [15, 16, 19]. Moreover, these cells circulate through the body without any immune or clearance risk that the NPs suffer, and they can easily infiltrate blood vessel barriers. Because of the innate features and their involvement in tumorigenesis, they are regarded as an ideal vehicle for drug delivery to realize the CAPIR cascade, as is shown in Figure 1(a).

### 2.1. Red Blood Cells (RBCs)

RBCs, also called erythrocytes, are the richest blood cell group. There are approximately 3.5–5 million RBCs per *μ*L, which have the longest lifespan of approximately 120 d. They also possess a high surface-to-volume ratio, and CD47 is expressed on the surface to protect cells from being taken up by immune cells. RBCs contain a large internal cavity without nuclei or organelles; thus, there are no normal endocytosis or exocytosis functions [22, 23]. RBCs contain approximately 270 million oxyhemoglobin molecules per cell, supporting their fundamental oxygen transportation function [24]. These features suggest that RBCs could be helpful as a carrier for drug delivery because they are easy to obtain, have a long circulation time with good biocompatibility and low clearance risk, are convenient for necessary modification, and have no possibility of tumorigenicity and a low drug leakage risk. Additionally, RBCs are oxygen-rich and can increase the productivity of toxic reactive oxygen species (ROS) for photodynamic therapy (PDT). This process enhances the PDT effect under a hypoxic tumor microenvironment and reduces PDT-caused O_2_ deficiency that boosts tumor growth [24].

### 2.2. Leukocytes

Leukocytes, formally known as immune cells, fight against diseases. Approximately 4000–10000 cells exist per *μ*L of blood, with at least a 24 h lifespan. When foreign substances, such as bacteria, enter the body, leukocytes respond to inflammatory signals and intrinsically chemomigrate back and forth through the blood vessel barriers to the diseased tissues. Leukocytes are part of the RES and can mobilize additional leukocytes to phagocytize particles or cross blood barriers. The ability of MAs to engulf aurum (Au) was increased 2.4-fold relative to that of nonphagocytes [25]. The unique engulfment, chemomigration, and immune activation features made them the perfect candidate as a drug carrier for target delivery.

#### 2.2.1. Monocytes (MOs)/Macrophages (MAs)

MOs are the largest blood cells and account for 2–8% of the leukocyte group. As a precursor, MOs are transformed into MAs once they are in tissues. They have versatile receptors on the cell membrane and react to foreign substances through nonspecific antigen recognition. Compared with other leukocytes, MOs/MAs responded to inflamed tissues rapidly and have the strongest ability for phagocytosis. They can be recruited to sites via several tumor-related factors: (a) cancer-related cytokines (e.g., CSF-1, VEGF, and PDGF); (b) chemokines (e.g., CCL-2/5/7/8/12); (c) fibrinogen; and (d) fibronectin and other factors produced during extracellular matrix (ECM) cleavage (in Figure 1(b)) [26]. After intravenous injection, it took MOs/MAs 6–12 h to arrive at inflamed tissues [27, 28] and in the brain [18]. Owing to chemohoming properties, MOs/MAs can penetrate the deep tumor matrix. Up to 70–80% of MAs were found in the tumor mass, part in the antitumor phenotype M1 and part in the protumor phenotype M2 [29, 30]. Having the largest size, a strong phagocytosis function, homing and penetration ability, and the possibility of the M1 antitumor phenotype make MOs/MAs beneficial for targeted drug delivery.

#### 2.2.2. Lymphocytes

Lymphocytes make up 25–35% of the leukocytes and are the smallest cells. They play an essential role in the immune response. Lymphocytes mainly include B, NK, dendritic cells, and T cells, in which T cells account for 75% of the total and work in the lymphatic fluid. Differing from the MOs/MAs, those lymphocytes activate an immune response via specific antigen recognition. Then, the activated cells present antibodies on the surface to specifically track and kill tumor cells through a ligand-receptor interaction [31]. EPR almost failed to function in some tumors, such as lymphomas, wherein the detected dose of either free drugs or NPs was 10 times lower than that in the blood, spleen, and liver. However, the activated polyclonal T cells can be successfully trafficked by tumor receptors, such as CD62L and CCR7, to the lymph node [12]. T cells were also recruited by CXCR4 and integrins *α*4, *β*1, and *β*2 to bone marrow and the spleen, respectively [12].

Similarly, NK cells can be chemoattracted by CXCL9 [17] and specifically recognize IL-2 on tumor cells [32]. Similar to MAs, T cells are another common cell type in tumor tissues [21], and it has been reported that T cells take 20–40 h to migrate to lymphoid organs in mice [12]. Based on specific recognition of tumor antigens, lymphocytes are normally used to activate the immune response of the patients to reduce the tumor burden. Moreover, because they patrol lymph nodes, lymphocytes carrying chemotherapeutics can simultaneously serve in both immunotherapy and chemotherapy to exert a cytotoxic effect on tumor cells.

#### 2.2.3. Neutrophils (NEs)

NEs are the largest leukocyte cell group, consisting of approximately 50–70%, and feature many internal NPs (0.2–0.4 *μ*m). Most particles are enzyme-rich lysosomes that are correlated with phagocytosis and digestive functions. NEs fight against foreign substances either through phagocytosis or neutrophil extracellular traps (NETs) [33]. Along with MOs/MAs, NEs possess strong innate chemotaxis with two kinds of chemokines: (a) collagen, fibrin fragments, products of activated complement, and cytokine and (b) microbial polypeptide with N-formylmethionine residue [34]. After interacting with chemokines, receptors, such as PSGL-1, CD44, and L-selectin, are highly expressed on the NE membranes [35]. Under inflammatory stimuli (IL-8, TNF-*α*, IL-1, and IL-17), the activated ECs overexpress E-selectin and P-selectin ligands to slow the NE rolling speed. The integrin superfamily (ICAM and VCAM) on the EC membrane further enhances the adhesion by binding with LFA-1 (*α*L*β*2) and Mac-1 (*α*M*β*2) on the NE surface [35, 36]. Additionally, Dietmar V is a shared and unique adhesion receptor related to transendothelial migration among different leukocytes [37]. A study showed that it took NEs 1 h to migrate to the stomach [38], and approximately 1.2–4.4% of NEs were in the tumor mass [39]. Moreover, an *in vitro* study showed that NP-loaded NEs could penetrate 80% of tumor tissues (*Φ* 300 *μ*m), yet NPs were only observed on the periphery [36]. The features, including a rich source, strong inherent phagocytosis, homing and penetration ability, and unique NETs formed under inflammatory conditions, make NEs a powerful carrier for targeting drug delivery [34].

### 2.3. Mesenchymal Stem Cells (MSCs)

MSCs are larger than the largest leukocytes and have a lifespan of approximately 1–2 d [19]. As adult stem cells, MSCs exhibit self-reproduction and multidifferentiation capabilities. They possess low immune rejection because of the nonspecific antigens on the cell membrane. MSCs also have a rich source, including blood, bone marrow, umbilical cord tissue, placenta, adipose tissue, and skin tissue. Identical to leukocytes, MSCs also have innate homing and migration ability to inflamed and tumor tissues. Tumor growth factors (e.g., EGF, PDGF-*α*, PDGF-*β*, HGF, and GDF-15), chemotactic factors (e.g., CXCL9 and CCL-25), matrix metalloproteinases (MMP1, MMP3, and MMP9), and inflammatory cytokines (IL-1*β*, IL-2, and IL-7) were discovered in liver tumors to chemoattract MSCs [19]. Additionally, the time MSCs circulate in the blood was reduced under diseased conditions, being 30 h in healthy mice, 24 h in mice with subcutaneous tumors, 18 h for orthotopically transplanted liver tumors, and 12 h in those with metastatic lung tumors [19]. However, an *in vitro* study confirmed that the migration ability of MSCs to breast cancer cells was 9 times higher than that of noncancerous cells [40]. Therefore, MSCs can actively and effectively track tumor tissues. In addition to the largest size, differentiation ability, low immunogenicity, rich sources, and chemomigration, MSCs additionally recruit and activate immune cells to tumor tissues [41]. Generally, MSCs show great potential as a carrier for targeting drug delivery.

## 3. Loading Strategies for Cargo Amounts and Cell Function Balance

Circulatory cells have been deployed to load varied cargos, including chemo/immunotherapeutic medicine (paclitaxel (PTX) [36], doxorubicin (Dox) [38], TRAIL [42], and siRNA [43]), radiotherapeutic agents (AuNRs [44], carbon nanotubes [45], ZnF16Pc [24], and Ce6 [46]), and diagnosis agents (fluorescent probe [47], ICG [48], and quantum dots [40]). The most commonly used loading methods are backpack and encapsulation. MOs were even reported to take an agent with a diameter of 7 *μ*m on the surface [49] and particles of 1 *μ*m inside [44] to cross the blood barrier that cargos alone cannot achieve. However, unlike inanimate NPs, cells respond to internal and external environments. Inappropriate loading approaches and cargo amounts may alter anticipated behaviors. Therefore, it is critical to balance the pros and cons on the premise of maintaining necessary cell functions.

### 3.1. Backpack Approach

The cell membrane, 7–8 nm thick, consists of a phospholipid bilayer as the basic skeleton, interweaved with proteins and glycolipids. The protein residues and oligo/polysaccharide chains on the membrane surface provide multiple possibilities to backpack cargos [50].

The backpack approach is simple, and cell preparation is not required. It is suitable for cells having special surface properties, such as releasing cargos via redox change [43, 51]; potential for *in vivo* cell binding; and easy regulation of the manner of cargo release. However, this approach has risks of detachment from the membrane, an alteration of membrane-related functions, or internalization by host cells.

#### 3.1.1. How to Conjugate Cargos on Membranes with Low Cell Function Impacts?

There are four cargo backpack methods. As shown in Figure 2, these include electrostatic/hydrophobic interactions [51], ligand-receptor binding via receptors on cell membranes [52], biotin-avidin binding via biotinylated cell membranes [53], and covalent conjugation via chemical groups, such as thiols or amines, on the cell membrane [54], wherein the biotin-avidin and covalent conjugation are considered the strongest binding and have specific ligand-receptor recognition that has the potential for *in vivo* hitchhiking use [55–57].

The cell membrane is essential for normal function, especially for the receptor-mediated signal pathways. Cargos attached to the cell membrane may influence cell behaviors, such as cell adhesion, migration, and even internal signal transduction [18]. Backpack place, cargo size, and loading amounts are important in this process. NPs attached to the main body exhibit a weaker impact on cell migration and reorganization than protrusion [58]. Additionally, NPs of 300 nm less than 100 ± 20 per cell did not substantially affect T cell function [54]. Likewise, using 5% of the cell membrane for Dox packing was acceptable; however, this means loaded drugs are 1.0 *μ*g per million cells [18]. Current free drug amounts of Dox [18], PTX [38], SN-38 [12], curcumin, and aPD1 [56] had a range of 1–3 mg per kg in animal tests and still showed limited therapeutic effects. Shp1 was demanded less, at approximately 76.5 *μ*g per mouse [59]. However, the cell amount used for clinical therapy was only approximately 1–10 million, although the recommended effective clinical dose is 4.58–11.92 mg per kg (Abraxane dose, calculated based on 60 kg, 175 cm patients) [60]. Rather than a burden, the cargo can therefore also be exploited to enhance rheotaxis. Gao et al. attempted to improve photosensitizer Ce6 backpack concentration and attain higher than 6 *μ*g mL^−1^, which caused RBC hemolysis within 48 h [46]. However, Tang et al. adopted another method to increase the amount without impacting cell functions. A negative charge surface was modified into a positive one and conjugated with anti-CD45 and IL-15Sa. The surface binding amounts were increased approximately 4-fold to 7.68 *μ*g per million cells [51].

Considering the necessary expected cell functions, the cargo density on the surface is a potentially involved factor, limiting the backpack amounts as were the NP properties [61]. Extra cargo modifications could weaken the impact on cargo conjugation and achieve an expected dose, such as receptors for recognition and cytokine loading for biological stimulation.

#### 3.1.2. How to Avoid Internalization?

Except for RBCs, both leukocytes and MSCs exhibit phagocytosis, which may threaten the backpack methods because cargos could be engulfed by carriers themselves [51]. To retain them on the cell membranes, factors related to the internalization process must be taken into account.

An early work by Jiang et al. indicated that internalization could be initiated by cell surface receptor-cytokine interactions [62], which Park et al. found was consistent on polystyrene sphere (PS). Compared with fibronectin-uncoated PS, the biocoated group increased internalization amounts by 3–5-fold [44]. Additionally, Li et al. modified NPs with the anti-CD73/90 antibody and found the loading amounts associated with MSCs increased 22% more than those of naked NPs [52]. Instead of a saturation-caused surface backpack, this may result from anti-CD73/90-enhanced internalization. However, receptor-mediated internalization does not necessarily mean initiation. Several receptors on T cell surfaces were reported to trigger the internalization process, yet the CD45a leukocyte common antigen on the cell membrane slowed the process. NPs modified with the anti-CD45 antibody could anchor on the T cell membrane for 6 h to several days to avoid internalization [51]. However, this differed for MAs because CD45 was internalized along with NPs [63].

Putting the receptor effect aside, the internalization process was also regulated by particle size. NPs of approximately 2–10 nm and 70–100 nm had a weaker initiation effect than those of approximately 25–50 nm on the process of receptor-mediated internalization of cancer cells [62]. Similarly, compared to 100–200 nm NPs, 50–100 and 200–300 nm NPs, respectively, had 1.56- and 2-fold lower uptake rates by MAs [64]. Both results exhibited a parabola tendency with a peak in the middle. This might be the optimal internalization size range, but it varies with cell lines because when the internalization process is slower than NP clustering on the cell surface, NPs would eventually not be engulfed [58]. This may further explain why internalized amounts of AuNPs were 1.5-fold lower with an increasing diameter from 7 to 14 nm [25]. A study by Park et al. on uncoated PS microbeads also indicated approximately a 2-fold decline of internalized amounts when size was increased from 100–200 to 1000 nm [44]. Although biocoating greatly enhances internalized numbers, the PS microbeads of 1000 nm internalized by MOs have strong phagocytosis ability and were only 1/800 of uncoated NPs of 45 nm engulfed by T cells [65]. Therefore, appropriately increasing NP size decreases the possibility of being internalized.

Other factors also influence the internalization process. Jiang et al. realized that this process could be greatly weakened at low temperatures [62]. Consistent with this finding, NP uptake amounts were decreased by 80% at 4°C compared to 37°C [18]. Based on this, Chandrasekaran et al. backpacked anti-CD57-modified NPs at 4°C to protect them from NK cell engulfment [42]. Huang et al. attached NPs at 4°C without antibody modification, and NPs were retained on the T cell surface for 3 d [12]. Moreover, some photothermal-therapeutic agents were cell-selective. Ly-6C^high^ MOs could internalize single-walled nanotubes (SWNT) to nearly 100%; however, for NEs, this was only 3%, and both Ly-6C^low^ MOs and lymphocytes were lower than 1% [45]. Another factor that influences the internalization process is NP shape. Nonspherical shape can decrease phagocytosis risk to some extent [49].

Generally, it appears that avoiding internalization-initiating receptor modification, increasing the NP diameter, lowering incubation temperature, and using a nonspherical shape may reduce the internalization risk. However, to what extent these factors influence and compromise cell functions in internalization progress still needs to be determined. An additional issue to be considered for the backpack approach is that NPs on cell membranes may cause protein corona formation, which could affect biological interactions because of the change in protein orientation and conformation [66].

### 3.2. Encapsulation Approach

Another cargo loading method, similar to the “Trojan horse,” was to encapsulate them into the inner cellular space, as shown in Figure 3. Normally, innate endocytosis was one way to engulf items, which can be realized simply by incubating cells and cargos together. However, it did not work for RBCs. Because of the lack of cellular organelles, RBCs lack the endocytosis function that leukocytes and MSCs have, such that hypotonic dialysis is always deployed in this condition.

The encapsulation approach provides possibilities for a high loading rate without altering the normal functions of cell membranes and for taking cargos through the blood vessel barrier without unnecessary interactions. However, it is also challenging because high loading rates increase the risk of cell cytotoxicity and unnecessary early leakage.

#### 3.2.1. How to Enhance Encapsulating Amounts without Cytotoxicity?

A high loading rate is one strong advantage of the encapsulation approach, but achieving this is quite complicated. Tumor chemotherapeutics/agents, such as PTX and Dox, are extremely toxic compared with the backpack approach, which was finished within 1 h. The encapsulation method always takes several hours to incubate the drug-loaded NPs or other agents with cells, as shown in Table 2. Consequently, there is the expectation that sufficient drug encapsulation will induce sudden cell death and therefore a low loading rate [18].

It was reported that 1–12.5 *μ*g mL^−1^ Dox was toxic to MAs [30, 67]. However, the Dox amounts that Fu et al. adopted were more than 4-fold, and no cell function effects were observed [68]. Except for MAs, Dox at such high concentrations also exhibited a small toxic effect on MSCs [52]. The two studies verified that most Dox-treated MAs and MSCs were in the G0/G1 phase; thus, they successfully escaped from the G2/M phase-dependent cytotoxicity of Dox. Additionally, drug-resistant protein P-glycoprotein was indicated on MAs [68] and MSCs [52] to facilitate Dox efflux and keep cells viable. The overexpressed ATP-binding cassette transporters on MSCs further maintained the stem cell state. Yet MSCs seemed more sensitive to PTX than Dox because 0.1 *μ*g mL^−1^ PTX was reported to be toxic to MSCs [69]. The discrepancy in Dox toxicity on MAs is still unclear because they have the same cell sources of RAW264.7. One deduction could be made: most of the MAs in the toxic groups were in the G2/M phase. One other finding was that placing Dox on NP surfaces instead of encapsulation resulted in 20% T cell death after 5 h and 60% after 15 h [70]. Thus, free drugs were not expected to be directly internalized by cells.

Strategies to solve this were to associate free drugs with NPs first and then encapsulate the drug-loaded NPs into cells to avoid direct exposure-caused cell toxicity. Several types of NPs that exhibited good biocompatibility, biodegradability, and capability to load hydrophilic/hydrophobic drugs were widely studied for drug carrying. Liposomes (including unilamellar and multilamellar) enhanced the maximum tolerated dose (MTD) 20-fold in MAs of PTX [71] and 50–200-fold for Dox [30, 67]. It was also reported that poly(lactic-co-glycolic acid) (PLGA) NPs were able to enhance 5-fold higher for Dox MTD for MAs [64], yet no obvious change was observed for PTX MTD on MSCs [69]. Huang et al. also deployed poly(AAc-co-DSA) and raised Dox MTD for MOs more than 3-fold [72]. One more drug-covering material is albumin. Albumin-bound NPs translated PTX into the commercial cancer drug Abraxane, for which the phase III data indicated that albumin allowed a 1.5-fold increase in MTD of Abraxane than that of free PTX; however, when the dose was beyond MTD, 25% of patients notably suffered from neutropenia [57]. Based on these findings, it is not difficult to conclude that encapsulating NP-protected drugs into cells prevents cytotoxicity and increases the loading rate.

#### 3.2.2. How to Ensure Retaining Sufficient Drugs Inside without Early Leakage?

Drugs are supposed to have a long retention period in cells. It took as long as 6–12 h for MAs to arrive at brain lesions [18], approximately 20–40 h for T cells to arrive at a lymphoid organ [12], and at least 4–6 h for MSCs to arrive at lung and liver tumors [19]. During circulation, drugs must stay with NPs to ensure the cell carrier function remains unchanged and there is sufficient drug for delivery to tumor sites. For example, 40% of Dox in NPs was released from MAs after 8 h [64], and 50–90% of SN-38 in NPs was released within 6–12 h [73]. It was also reported that approximately 60% of PTX in NPs was released from MSCs within 30 min [74]. These facts indicate that most drugs were unloaded before arriving at tumor lesions and further cause systematic toxicity.

One leakage threat was from lysosomes. This organelle has a low pH of 5 and is flooded with approximately 60 types of hydrolases, which may degrade NPs inside the organelle. Acid-responsive NPs were found to begin intracellular release within 15 min [75]. Therefore, the backpack approach is suggested to carry unprotected, acid-responsive drugs/NPs for cancer therapy. Another threat was from exocytosis. Cells engulfed drugs/NPs inside via endocytosis, but exocytosis correspondingly placed encapsulated NPs in danger of leakage. Interestingly, the two threats are not related to RBCs because they do not have lysosomes or an exocytosis function. RBC membranes are impermeable, and normally, no more than 5% of free drugs leak within 2 h [46]. Besides lysosomes and exocytosis, drug-resistant protein P-gp is one more threat for cells that expressed the protein because it was found that 65% of free Dox was extruded from MAs within 2 h [68].

One option is choosing proper NPs that are themselves beneficial for drug retention to reduce leakage risk. For example, poly(AAc-co-DSA)-coated Dox has a restricted release lower than 20% within 24 h from MOs [72]. Another solution is modulating NP structure. Instead of polymers or liposomes, Zhang et al. adopted silica as a nanocapsule to load Dox and then encapsulated the complex into MAs [18]. To realize minimal liberation during migration and controlled release *in situ*, the drug-loaded MAs achieved a two-phase drug release by modulating silica coating thickness from 12 to 52 nm and keeping two times the amount of the drugs inside NPs. One more possibility is to enhance the internalization process, which was discussed in detail in Section 3.1.2. Based on this strategy, Moku et al. attached one cell-penetrating peptide-transactivator of transcription (TAT) peptide on the cell membrane. Compared with naked NPs, the uptake of TAT NPs was enhanced 3-fold, and retention amounts of drugs/NPs were accordingly increased 2-fold in MSCs, as expected [74].

## 4. Cascade Strategies for Improving Cell-Driven Targeting Delivery Efficiency

The delivery efficiency of NPs varied with tumor types, targeting methods (active or passive), material properties (inorganic/organic, particle size, surface charge, and particle shape), and transplantation approaches (orthotopic allo/xenografts). The factors mentioned above strongly affect the delivery efficiency and have been well studied for NPs. However, according to the analysis of over 10 years (2006–2016), the delivery efficiency of NPs to tumors was still less than 1%, with only 0.7% reaching the lesion on average, and the majority was in a nonspecific interaction manner [10]. This low delivery efficiency in tumors resulted from the following facts: NPs were cleared by RES and kidneys [8]; NPs rely on EPR effects to accumulate in tumor lesions, which failed in the clinic [76]; and a 10-40-fold fluid interstitial pressure hampered NP penetration and distribution [10]. Recently, circulatory cells from the blood were widely studied, as listed in Table 3, which shows great potential to facilitate the CAPIR process to improve diagnosis and therapeutic efficacy.

### 4.1. Circulation Ability

Regarding clearance threats on NP-based DDS, the long circulation time of circulatory cells in the whole body, as discussed in Section 2, reduces the risk to an extremely low level. In the study of Huang et al., 60% of Dox/NP-encapsulated MOs arrived in prostate tumors after 48 h postintravenous injection, but 80% of free NPs were found trapped in the liver [72].

### 4.2. Accumulation Strategies

The concern about the EPR-dependent accumulation of NPs would not hinder circulatory cells because they are chemoattracted by tumor-related signals and actively transmigrated into tumors with their payloads. However, a recent study found that, instead of long-term recognized intercellular extravasation, NPs deployed an active transportation manner via transcellular mechanisms to accumulate into tumor tissues [9]. The work revealed that gap frequency was as low as 8% in all studied tumor types, in which more than half the gaps were transcellular channels. Would it be controversial that NPs were difficult to accumulate in tumors without obvious EPR effects? If not, did it result from low retention, despite being transported inside? Regardless of whether NPs depend on EPR or not, they must face the same issue of the low accumulation rate that circulatory cells can enhance. Based on the following three strategies, accumulation of the cell vehicle was achieved, and the efficiency was enhanced.

#### 4.2.1. Innate Homing Ability

The basic approach to target the lesion was based on the innate chemotaxis response of cells to tumor-related signals, as depicted in Section 2. Compared with the average mentioned above that reached a rate of 1%, approximately 44.4 ± 5.4% of PTX/NP-encapsulated MSCs arrived in mouse gliomas through natural homing ability [69]. Dox/NP-encapsulated MA-treated mice also appeared to have a higher density in glioma tissue than Dox/NP alone [64]. The accumulation amounts of SN-38/NP-backpacked T cells were 63 times higher than that of free SN-38/NPs at 20 h in lymphomas and remained high for 4 d [12]. It was confirmed that several ligand-receptors bound to blood vessels could slow the rolling pace of cells and facilitate the transmigration process [35]. Similarly, Chen et al. revealed that ECs in tumor vasculature had different phenotypic profiles with various shear stresses, and ligand-receptor interaction can resist the flow stress and extend residence time on EC surfaces, thereby increasing the accumulation rate [14].

#### 4.2.2. Amplifying Tumor-Related Signals *In Situ*

One method to improve accumulation rate is to amplify the inflammatory tumor signal for chemoattraction based on innate homing ability:

- Under a postsurgical inflammatory condition, Xue et al. increased the targetability of PTX/NP-encapsulated NEs 86-fold and 1162-fold compared to that of PTX/NPs and single Taxol, respectively [36]
- Radiation is also employed to enlarge local inflammatory conditions. Using enhancing radiation intensity, inflammatory factors such as IL-8, IL-10, and TNF-*α* in tumors were amplified approximately 1.3–1.56-fold. Accordingly, NEs exhibited a radiation dose-dependent tumor accumulation, showing obvious cell clusters in tumors at 1 h postinjection, which lasted for 2 d [38]. After *γ*-ray pretreatment, a hypoxia core featured by a decreased vascular density and increased hypoxia microenvironment was augmented in tumors to recruit tumor-associated MAs. In this context, Dox/NP-encapsulated MOs presented a higher aggregation in tumors than did Dox/NPs [72]

#### 4.2.3. Targeting Modification on Cell Carriers

Modifying cells themselves is another method to support high accumulation rates:

- Lymphocytes can recognize tumors via specific antigens; therefore, they retain tumor-related antigen receptors and facilitate this process. For example, NP-backpacked CD8+ T cells retained receptors that specifically recognized OVA-1 in tumors, which amplified accumulation 176-fold more at the tumor site than free NPs after 2 h [54]. Engineered NK cells that expressed CD19 and Her2 receptors showed higher accumulation rates than nonengineered cells against CD19/Her2-positive tumors [17]. Recently, cytotoxic T lymphocytes were reported to release supramolecular attack particles (SMAPs) with TSP1 surface proteins to target tumor cells and then performed independent killing [77]
- Conjugating targeting molecules on the cell surface. RGD is a short peptide that targets *α*v*β*_3_ integrin-positive tumors, and modifying RBCs with RGD allowed an obvious attachment in tumors that native RBCs could not achieve [23, 48]
- For magnetizing modification, cell carriers have internalized magnetic particles, such as Fe_3_O_4_, to follow guidance from electromagnetic fields. This method was widely studied as external assistance to control the cell path, and MA motion and speed were found to be enhanced 29 times that of normal cells [71]. Along with this, it may improve SMAP capability and make a concession to the premise of reducing early leakage risk

Enhancing accumulation can reduce drug demands. SN-38/NP-backpacked T cells had density 90 times higher in lymphomas than that in free drugs of 10-fold injection doses. Moreover, T cells with a 1/40 drug dose of free SN-38 eased the tumor burden that free SN-38 could not [12]. It was also found that TNF-*α*-transduced MSCs secreted TNF-*α* for 2 weeks and showed equal effects at a low dose to free TNF-*α* at a high dose [41].

### 4.3. Penetration Ability

NPs normally are distributed around the periphery of tumor tissues. For example, Dox was reported to diffuse only 8–16 *μ*m from the tumor vessel, and Dox/NPs were limited to 10–20 *μ*m [72]. By modulating NP size, infiltrating long distances could be feasible. NPs can penetrate into deep tumor tissue only if the diameter is smaller than 20 nm, and this size range will be difficult to escape from RES clearance [4].

Unlike NPs, circulatory cell-driven drug delivery was able to chemomigrate without obstacles even under the condition of a high-pressure tumor matrix. As discussed in Section 2, leukocytes and MSCs are components of tumor tissues. Furthermore, leukocytes can perform compartmentalized and mixed distribution in tumors [78]. In animal tests, it has been confirmed that, regardless of high pressure, the hypoxic microenvironment in the tumor tissues had a stronger ability to recruit leukocytes into deep regions [72]. In glioma, spheroids at the depth that Dox/NP-MAs migrated were 1.56-fold that of NPs alone (56.42 *μ*m vs. 36.07 *μ*m) [64]. Furthermore, Dox/NP-MOs penetrated farther than 100 *μ*m from the nearest vessel [72]. Therefore, once drug-carrying circulatory cells accumulated in the tumor sites, the penetration process was in a clear pattern.

### 4.4. Drug Release Profiles and Internalization

Concerning the CAPIR cascade, the final two steps of NPs were internalization for drug release, but the order for circulatory cells was reversed. Cargos were released first via transcellular mechanisms, then were internalized by tumor cells. As illustrated in Figure 4, there are three kinds of drug release patterns for cell-driven drug delivery systems, as discussed below.

#### 4.4.1. Exocytosis

Exocytosis was the fundamental function that drug-encapsulated cells employed. By optimizing the drug leakage profile during circulation, drugs/NPs released via exocytosis could be slowed in the early phase and quickened in the late phase for tumor cell internalization [18]. Drug efflux also occurred after the drugs and NPs were dissociated inside cells [69]. This meant that drugs/NPs were internalized by tumor cells in two patterns: intact drugs/NPs and free drugs.

The internal tumor microenvironment was also reported to accelerate exocytosis speed. Under inflammatory signals of the IFN-*γ* condition, Dox/NP-MAs were activated to release the drug two times faster within 4 h than the group without IFN-*γ* [64]. The same tendency happened to Dox/NP-MOs in acidic tumor environments [72]. However, exocytosis did not work for RBCs because there are no organelles to function in efflux, and they rely on diffusion or disintegration only.

#### 4.4.2. Cell Disintegration

Cell disintegration was one pattern to trigger drug release in lesions, used for both the drug-encapsulated and backpacked cells. As mentioned in Section 3.2.2, chemotherapeutics threatened the normal function of cells. When they arrived at the tumor sites, free drugs reached a high concentration inside carriers as designed, and cells started to disintegrate to release all tumor-toxic freights [30]. Additionally, NEs had a unique feature that could amplify this toxic process. Under a condition of high postsurgical inflammation environment of TNF-*α*, CXCL1/KC, and IL-8, NEs could destroy themselves into NETs to release both original toxic proteins and loaded toxic drugs [36].

External interventions like ultrasound, radiation, heat, and NIR were also deployed to destruct cells for drug release *in situ*. Those interventions were initially involved in radiotherapy. With ultrasound aid, MOs encapsulated with echogenic particles and drugs disintegrated and showed substantial cancer cell killing ability *in vitro*. RBCs released 80–100% of Dox under radiation conditions within 10 min, and the speed was 16 times faster [23, 46]. RBC disintegration is an important premise for PDT, which can simultaneously damage tumor vasculatures and generate abundant ROS toxic to cancer cells [24]. However, additional approaches are united for chemo/radiotherapies and diagnoses to amplify treatment efficacy. Suppose both imaging agents and photosensors are carried via RBCs and can simultaneously realize bioimaging-directing tumor resection via NIR-II fluorescence and killing tumor cells under the PDT condition [48]. Given the disintegration-responsive feature under acidic environments and NIR laser conditions, MAs released 29.3 ± 1.69% of the drugs in 1 h, which took approximately 24 h under a pH of 7.4 with no laser conditions [67].

#### 4.4.3. Cell-Drug Dissociation

Cell-drug dissociation is another pattern to unload cargos into the tumor sites. For these drugs that cannot interact with tumor cells well if retained on the host cell membrane, cell dissociation must be considered. Li et al. backpacked MSCs with Dox/silica nanorattles that were responsive to pH change. Compared with pH 7, pH 4 led to an alteration of interaction force strength between nanorattles and drugs and stimulated a 3-fold greater dissociation [52]. Similarly, Tang et al. backpacked T cells with a protein nanogel interlinked by a reduction-responsive reversible cross-linker. Once in tumor tissue, the raised tumor antigen concentration activated T cells. The surface reduction was correspondingly increased on the cell membrane, which initiated cell dissociation with drugs [51].

#### 4.4.4. Internalization and Survival Extension

Regardless of adopting any release approach, drugs/NPs were internalized in a mixed manner for free drugs and drugs/NPs, except for those products, such as ROS, performing killing tasks completely without internalization. The internalization efficiency of drugs/NPs in tumor cells was determined by NP design, and carrier cells hardly played a role in this process.

The cell-driven drug delivery system at least extended the survival rate. After tumor surgery, the number of survival days of SN-38/NP-T cell-treated mice was extended by 10 d relative to both free SN-38 and SN-38/NPs [12]; that of Shp1/NP-T cell groups showed a 14 d increase compared to that of the untreated group [59], and that of PTX/NP-NE-treated mice was, respectively, increased by approximately 32 and 23 d longer than free Taxol and PTX/NPs [36]. In general, these targeting strategies with circulating cells pragmatically overcame the problems NP-based systems faced. Regardless of some issues to be solved, such as balancing loading amounts and function, it created new strategies and insights for targeted cancer therapy.

## 5. Cell Derivatives as Drug Carriers for Targeting Delivery

As biological entities, native cells are complex and fragile. Augmenting while balancing the functionality remains a topic of study. Two other candidates derived from cells provided extra clues for targeting drug delivery: the cell membrane and small extracellular vesicles (EVs), as listed in Table 4.

### 5.1. Cell Membrane

#### 5.1.1. Native Cell Membrane

The efficiency of circulatory cell delivery of drugs is attributed to the following features: reducing RES clearance risk, targeting and accumulating in tumor sites, and exerting a cytotoxic effect. These topics have been partly related to cell membrane proteins that provide a “do not eat me” signal [22], tumor-targeting proteins [46], and death-initiating proteins [77]. Therefore, the cell membrane plays a key role in drug/NP delivery.

Cell membranes of circulatory cells are biological materials. As expected, they present good biocompatibility, long circulation time, and tumor-targeting and accumulation abilities. Blood leukocyte membranes express signature protein CD45 or CD3Z and adhesion protein LFA-1 or CD11a for vascular extravasation [79]. NK membranes express the signature protein CD56 and tumor-targeting/toxic receptors NKG-2D and NKp30 [32]. After being used to decorate NPs, leukocyte membrane- and NK membrane-coated NPs were stable in both PBS and 90% fetal bovine serum within 24 h, and no early degradation or drug leakage was observed. However, the membrane-coated NPs presented a donor membrane-dependent clearance where particles exhibited the same membrane as phagocytic cells, and the internalization chance decreased by approximately 75%. When this does not occur, it is low to 10% [79]. Both kinds of membranes facilitated a 2-fold higher accumulation in tumors relative to that in free NPs. Consistent with this, MA membrane-coated NPs reached a mean retention time and half-life in the plasma 2 times more than that in uncoated NPs [80]. MA membranes were additionally found to have 5.88-fold higher cellular uptake efficiency than that of uncoated NPs [81]. Unlike the top-down approach in the studies mentioned above, Parodi et al. functionalized particles with leukocyte lesion-targeting molecules to create a leukosome via the bottom-up method. Compared with naked particles, it also decreased clearance from RES and kidneys by 1.5–2.6-fold and increased accumulation 7-fold in the inflamed vessels [82]. In addition to leukocytes, membranes of RBCs [83], platelets [84], and stem cells [85] were also widely used for particle camouflage. Cancer cell membranes were also studied as NP coating to target cancer cells in return. Compared with naked NPs, liposome-coated NPs, RBC membrane-coated NPs, and trypsinized HeLa membrane-coated NPs, HeLa membrane-coated NPs achieved enhanced cellular uptake efficiency [86]. This did not necessarily mean the cancer cell membrane itself surpassed other membranes to target tumor cells, because one cancer-specific membrane protein on the HeLa cell-integrin *α*v*β*3 was found to function in HeLa targeting. Therefore, the tumor-targeting design should be based on distinct cancer cell types.

#### 5.1.2. Synthetic Membrane/Cell

By mimicking the natural function of cell carriers, synthetic membranes and cells were constructed. Because hemoglobin itself is susceptible to autooxidation, to overcome large oxygen loss for PDT, Liu et al. assembled artificial RBCs with basic features of size, shape, and deformability. Amazingly, the artificial RBC capacity was augmented to achieve 10-fold payloads of a hemoglobin-dopamine complex [87]. Similarly, Guo et al. deployed a silica cell bioreplication method to rebuild RBCs successfully, and these cells expanded possible carrying contents from hemoglobin to drugs, ATP biosensors, and magnetic NPs [88]. Hindley et al. deployed a bottom-up synthetic strategy to behave biologically to construct an artificial cell with a communication pathway [89]. Strictly speaking, a synthetic cell/cell membrane is not a cell derivative, especially for synthetic cells similar to a robot, which is a simplification and augmentation process that screens unnecessary functions and amplifies/adds expected ones. However, they provide a new perspective on the DDS beneficial elements from cells.

### 5.2. Small Extracellular Vesicles (Small EVs)

#### 5.2.1. A Real Drug Delivery Medium *In Vivo*

Extracellular vesicles are lipid bilayer-coated and are released from parent cells, consisting of small extracellular vesicles of exosomes (30–150 nm), ectosomes (100–1000 nm) [90], large vesicles of apoptosis bodies (1–5 *μ*m) [91], and oncosomes (1–10 *μ*m) [92]. These vesicles have versatile contents, including proteins and genetic materials, secreted for short/long-distance communication by all types of cells under physiological and pathological conditions. EVs have rich sources in body fluids, such as blood, saliva, urine, cerebrospinal fluid, and milk.

Small EVs are involved in drug delivery *in vivo*. Smith et al. found that carbon nanotubes were taken up by 8 *μ*m circulating cells once injected into the blood [45]. Recently, Chaudagar et al. observed a similar phenomenon wherein NEs were *in vivo* activated to internalize NPs (BSA-NP-cabozantinib) to assist drug delivery to lesions [55]. Kim et al. further realized that, instead of being internalized directly by tumor cells, NPs could be first engulfed by local MAs [93]. Importantly, approximately 16.5% of released drugs were entrapped within MAs-exosomes by calculation [18]. More recently, it was revealed that cytotoxic T lymphocytes killed cancer cells by releasing both ectosomes and supramolecular attack particles, wherein supramolecular attack particles were found to work independently [77]. Because NPs are taken into mediating cells and entrapped in vesicles, studies have paid much attention to small EVs as carrier candidates.

#### 5.2.2. Carrier Features of Small EVs for Drug Delivery

Besides a nanoscale size similar to that of NPs and blood circulation properties similar to those of circulatory cells, small EVs also provide targeting efficiency and have the potential to reduce cell carrier side effects. Similar to cell carriers, the loading method is a critical link for small EVs, and it has been detailed elsewhere by Yang et al. [94]:

- Small EVs have an inherent escape capability from clearance. Ectosomes of RBCs were reported to maintain the parent “don't eat me” protein CD47 [22]. Yang et al. then utilized blood exosomes for delivering Dox, which reduced drug accumulation in the liver and heart [95]
- Small EVs were able to target and accumulate in tumor tissues as cells did. EVs contained transmembrane signature proteins and versatile receptors for membrane anchoring. For example, except for T cell signature proteins of CD8 and CD3, exosomes and ectosomes were shown to retain tumor-targeting proteins of T cell receptors (TCRs) [96] and FasL, respectively [77]. Both proteins can initiate tumor death. Moreover, the amounts of surface chimeric antigen receptors (CAR-engineered tumor-targeting proteins) on purified exosomes were similar to those on cells [96]
- Inflammation and low pH are two hallmarks of the tumor microenvironment. As discussed in Section 2, inflammatory signals chemoattract related cells to sites and enhance the EV internalization process. TNF-*α* loosened the tight conjunction between cells, and the activated cells had 3 times higher internalization ability with a time extension [97]. A low pH value also increased the timing of exosome uptake by tumor cells. Under acidic conditions (pH 6), the uptake emerged 15 min earlier than that under a pH 7.4 condition, and the uptake amounts were 1.5-fold higher during the first 5 min [98]. An acidic environment further increased cargo release efficiency. Instead of being engulfed into lysosomes, exosomes under acidic conditions tended to directly fuse with the tumor cell membranes to release the cargo. It was also shown that the fusion process was cell-dependent. The fusion activity of tumor exosomes was 19–23% for metastatic tumor cells and 9–12% for primary tumor cells, whereas it was barely detectable in normal cells, which provided another perspective on exosome targetability
- Small EVs can reduce cell carrier side effects while efficiently killing tumor cells. An important feature of CARs-exosomes inherited from cytotoxic T cells is that they can exert a cytotoxic effect against tumor cells. Additionally, CARs-exosomes perfectly rid themselves of PD-1 on the vesicle membrane (PD-1 is normally expressed on parent cells and interacts with PD-L1 on the tumor surface to weaken the cell antitumor effect). No cytokine release syndrome was observed in CAR-exosome therapy, common toxicity in CAR-T therapy [96]

#### 5.2.3. Application of Small EVs in Tumor-Targeting Delivery

Small EVs secreted from donor cells retained the mother cell signature and function protein, and the selectivity was maintained, to some extent, to ensure targetability and therapeutic effects.

Exosomes from engineered leukocytes expressed tumor-targeting Lamp2b, which reached an encapsulation efficiency of 20% with Dox. Dox/EVs appeared in tumor sites within 30 min after injection, peaked at 2 h, and disappeared at 8 h, although no signal was detected in the tumor area at any time for nontargeting protein exosomes [99]. The off-target case in the control group may be caused by losing some of the tumor-targeting proteins of donor cells. CAR-T-derived exosomes retained the necessary targeting proteins and inhibited 67–70% of tumor growth for both the breast and lung cancer therapies in animals [96]. Another study showed the same tendency [100]. Instead of bioengineering, Wang et al. fed donor cells with PTX and biotinylated these cells, then obtained expected PTX-loading exosomes with dual ligands of biotin and avidin on the membrane to target tumor cells. These biotinylated exosomes extended the accumulation signal to 48 h after injection, but blank exosomes were almost lost in circulation. This loss may result from cell line discrepancy because circulatory cells (usually leukocytes) were the ones with rich tumor-related targeting proteins. Dumontel et al. interestingly used tumor cell-derived exosomes to encapsulate ZnO nanocrystals and effectively kill tumor cells without any membrane modification [101]. Magnetic molecules were also applied to small EVs for targeting. Zhan et al. linked Fe_3_O_4_ nanoparticles on blood exosomes via a ligand-receptor interaction to simultaneously achieve both exosome separation and tumor targeting. The magnetic exosome group enhanced vesicle accumulation at the tumor site within 1 h to a level that the normal group took 24 h to achieve (Figure 5) [102].

Besides chemotherapeutic drugs, genes are another type of cargo that have been widely studied with small EVs. One advantage, as discussed previously, is that small EVs can fuse with cell membranes directly to prevent genes from degradation in lysosomes. Additionally, because of the lack of nuclei and organelles in RBCs, RBC-derived microvesicles are a great carrier for gene delivery. Usman et al. deployed RBC microvesicles to load antisense oligonucleotides to successfully treat leukemia [103]. To cross the endosome membrane, endosomolytic peptide L17E was tethered on EVs to accelerate the escape of cargo from endosomes to the cytosol. Compared with nonmodified exosomes, RNA in modified exosomes that was entrapped in endosomes was less than one-third [102].

These EVs displayed a prolonged circulation time, high targeting efficiency, and therapeutic effects by modulating membrane protein expression and cell line discrepancy between donors and target cells. A clinical finding regarding methotrexate-containing microvesicles for treating cholangiocarcinoma reported that approximately 30% of patients were partially relieved upon biliary obstruction. After the first treatment, approximately 50% of the liver function of the patients was improved, and symptoms of jaundice were reduced [104]. This suggested the feasibility of small EVs as a competent drug delivery carrier for tumor therapy.

## 6. Challenges

### 6.1. Restricted CAPIR Process

There are two concerns regarding RBC accumulation and penetration ability. A high surface-to-volume ratio causes high deformability, yet it matters to what extent cells of 7–8.5 *μ*m can transmigrate the 2 *μ*m interendothelial gaps. Moreover, these cells are passively driven by blood flow, so they may have a problem penetrating the deep tumor matrix alone.

Similar to RBCs and cell membranes, crossing the blood barrier and accumulating well is a persisting issue for EVs because they cannot migrate as leukocytes/MSCs do. One *in vitro* Transwell study reported that exosomes migrated from a low chamber to an upper one via a transcellular mechanism [97] instead of gap diffusion. Sindhwani et al. recently also revealed that only seven EPR gaps were found in 313 vessels [9]. When taking the transcellular way, both the uptake-to-efflux ratio and the integrity of EVs need to be determined, because an inflamed endothelium with highly expressed adhesion molecules and inflammation factors facilitate EV internalization, similar to ICAM-1 and TNF-*α* [105]. Additionally, the penetration ability of nano-EVs such as NPs may be weaker than that of cells under high fluid interstitial pressure, which impacts the distribution of EVs in lesions and the drug delivery efficiency afterward.

One addition that should be taken into consideration is that, to some extent, drugs loaded by cells increased survival rates, but attention has to be paid that it cannot completely prevent the regrowth of tumors, although it efficiently slows tumor recurrence [36].

### 6.2. Bringing New Issues

The demands of drug-loaded leukocytes were 10 times more than the normal level, which might evoke side effects in blood and obtain a great number of cells from patients themselves [106]. Additionally, the therapeutic effects of leukocytes were dependent on the *in situ* inflammatory level—no inflammation signal and no specificity [36]. Leukocyte-based therapies were further determined to cause two unique toxicities: cytokine release syndrome and immune activation syndrome [96], with a risk of secondary malignancies [68]. The clinical trial data of FDA-proved anti-CD19 CAR-T cell therapies indicated an association with B cell malignancies in 50–90% of patients [96]. Not only did leukocytes have secondary malignancy risks, but stem cell-based therapy also revealed a tumorigenicity possibility [107], which was immune-dependent [41]. Stem cells even partially contributed to the recruitment and activation of immune cells to tumor tissues and partially facilitated metastasis [19].

## 7. Conclusion

In recent decades, increasing efforts have focused on cell-driven drug delivery systems in the tumor area. Most of these were circulatory cells because they had special characteristics that the CAPIR cascade required, but NP-based DDS alone could not achieve to date, such as inherent biocompatibility, long circulation time, active accumulation, high penetration ability, and immune response activation. Despite emerging challenges, cell-driven drug delivery systems have performed well to date in enhancing targeting delivery efficiency. Clues for resolving the current limitations of the NP-DDS were encountered and provided the possibility for the development of precision medicine for cancer diagnosis and therapy.

## Figures and Tables

**Figure 1:** (a) Scheme of the CAPIR cascade of a nanomedicine to deliver a free drug into cancer cells. The overall efficiency, *Q*, is the product of the efficiencies of five steps. Reproduced with permission [4]. Copyright 2017. John Wiley and Sons. (b) Overview of molecules that can recruit monocytes/macrophages to tumor sites and turn into tumor-associated macrophages. Reproduced with permission [26]. Copyright 2009. John Wiley and Sons.

**Figure 2:** (a) Scheme of NPs conjugated with cell membranes via electrostatic interaction. (b) Dox was bound on the MSC membranes via the CD90/CD73 antibody-ligand interaction. Reproduced with permission [52]. Copyright 2011. American Chemical Society. (c) FluoSpheres (red) modified by NeutrAvidin (orange) to bind to biotinylated MSC membranes. Reproduced with permission [58]. Copyright 2010. American Chemical Society. (d) SN-38 NPs were anchored on T cells via a thiol group expressed on the cell membrane. Reproduced with permission [12]. Copyright 2015. American Association for the Advancement of Science.

**Figure 3:** Backpack and encapsulation approaches. (a) Scanning electron microscope (SEM) images of RBCs which were backpacked with multitheranostic probes for cancer surgery guidance and therapy. (b) SEM images of higher magnification of cargo-loading RBCs, and the insert shows naked RBC images. Reproduced with permission [48]. Copyright 2019. Ivyspring International Publisher. (c) Confocal micrographs of quantum dot distribution in MSCs after 15–30 min, 1 h, 6 h, and 24–48 h incubation. Nuclei, Hoechst blue; actin, Phalloidin green; quantum dots, red. Scale bar for main images, 15 *μ*m; scale bar for insert images, 10 *μ*m. Reproduced with permission [40]. Copyright 2017. Dove Medical Press.

**Figure 4:** Three drug release patterns. (a) Exocytosis: either free Dox or Dox/SiO_2_ NPs were secreted by MAs for glioblastoma treatment. Reproduced with permission [18]. Copyright 2018. John Wiley and Sons. (b) Cell disintegration I: Abraxane-encapsulated NEs disintegrated and formed the neutrophil extracellular traps to kill gastric cancer. Reproduced with permission [38]. Copyright 2018. John Wiley and Sons. (c) Cell disintegration II: Dox-encapsulated and Ce6-backpacked RBCs were disintegrated by photoradiation for breast cancer. Reproduced with permission [46]. Copyright 2017. American Chemical Society. (d) Cell-drug dissociation: SN-38 was dissociated from the T cell membrane into lymphoma cells. Reproduced with permission [12]. Copyright 2015. American Association for the Advancement of Science.

**Figure 5:** (a) Scheme of gene/chemotherapy on a blood exosome basis. Chemotherapeutic drugs and the cholesterol-modified miRNA21 inhibitor were embedded between the vesicle lipid bilayers for tumor killing; both magnetic molecules and L17E peptides were bound onto the vesicle membrane, respectively, for targeting and lysosome escape. (b) According to nanoparticle tracking analysis (NTA), the original exosome size was 93 nm. (c) The size was increased to 106 nm on average, after cargo loading and membrane modification, and transmission electron microscope (TEM) images showed modified exosomes that retained a clustered structure. Reproduced with permission [90]. Copyright 2020. Ivyspring International Publisher.

**Table 1:** Properties of red blood cells, mesenchymal stem cells, and leukocytes.

	RBC	MSC	Leukocyte					
Amount (million/*μ*L)	3.5-5	To be determined	0.0004-0.001					
			Neutrophil	Eosinophil	Basophil	Monocyte	Lymphocyte	
			50-70%	1-3%	0.4-1%	2-8%	25-35%	
							T cell	B cell
							75%	10-15%
Diameter (*μ*m)	7-8.5	30-40	10-12	12-15	12-15	20-30	6-12	6-12
Lifespan (days)	120	1-2	3-4	8-12	12-15	1-5	4-35	>30

**Table 2:** Cargo loading conditions of encapsulation and backpack approaches.

Refs.	Loading method	Culture time	Incubation temperature	Drugs/NPs	Drug/NP size (nm)	Drug concentration for loading	Cell carrier type	Final loading amounts (*μ*g drug per million cells)	Cancer type	*In vitro*/*in vivo*
[70]	Encaps	5 min	Unknown	Dox/TargetMAG NPs	50	2 *μ*g/mL	T cell	Dox 0.192	N/A	*In vitro*
[18]	Encaps.	2 h	37°C	Dox/silica NPs	28.4	20 *μ*g/mL	MA	Dox 16.6	Glioma	*In vivo*
[72]	Encaps.	4 h	37°C	Dox/poly(AAc-co-DSA) NPs	260	13.6 *μ*g/mL	MO	Dox 1.44	Prostate cancer	*In vivo*
[67]	Encaps.	6 h	Unknown	Dox/liposome NPs	145	25 *μ*g/mL	MA	Dox 4.4	Breast cancer	*In vivo*
[69]	Encaps.	8 h	37°C	PTX/PLGA NPs	135	8 ng/mL	MSC	PTX 1	Glioma	*In vivo*
[38]	Encaps.	12 h	Unknown	PTX/albumin NPs	100-130	200 *μ*L PTX	NE	PTX 18	Gastric cancer	*In vivo*
[53]	BP	20 min	Unknown	Curcumin/chitosan NP-biotin	377	50 *μ*g/mL	MSC	Curcumin 54.73	Lung cancer	*In vivo*
[59]	BP	30 min	37°C	NSC-87877/liposome NP-PEG	200	T cell : NP ratio = 1 : 1000	T cell	100 NPs/cell	Prostate tumor	*In vivo*
[12]	BP	30 min	4°C	SN-38/liposome NPs	340	Unknown	T cell	SN-38 0.4	Lymphoma	*In vivo*
[46]	BP	30 min	RT	Chlorin e6	Molecule	3 *μ*g/mL	RBC	~6 × 10^6^ Ce6 molecules on the surface	Breast cancer	*In vitro*
[51]	BP	1 h	37°C	IL-15Sa/nanogel-PEG	121	0.67 *μ*g/mL	T cell	IL-15Sa 7.68	Melanoma	*In vivo*
[52]	BP	1 h	37°C	Dox/SN-anti-CD90/CD73	152.9	100 *μ*g/mL	MSC	1500 NPs/cell	Glioma	*In vivo*
[24]	BP	1 h	4°C	ZnF16Pc/biotin-ferritin	15-18	Unknown	RBC	2 × 10^7^ ZnF16Pc molecules on the surface	Glioma	*In vivo*

Encaps. = encapsulation; BP = backpack; RT = room temperature. For other abbreviations, please refer to the abbreviation list.

**Table 3:** Different cells loaded with varied cargos for cancer diagnosis and therapy.

Refs.	Cell type	Loading method	Drugs/NPs	Drug/NP size (nm)	Cancer type	*In vivo*/*in vitro*
[36]	NE	Encaps.	PTX/liposome NPs	100	Glioblastoma	*In vitro*
[38]	NE	Encaps.	BSA/PTX NPs	130	Gastric cancer	*In vivo*
[55]	NE	Injecting and engulfed by NE *in vivo*	BSA/PLGA NPs	450	Prostate cancer	*In vivo*
[12]	T cell	BP	SN-38/liposome NPs	340	Lymphoma	*In vivo*
[43]	T cell	BP	siRNA/liposome NPs	150	N/A	*In vitro*
[59]	T cell	BP	NSC-87877/liposome NPs	200	Prostate cancer	*In vivo*
[51]	T cell	BP	IL-15Sa/nanogel	121	Melanoma	*In vivo*
[54]	T cell	BP	Liposome NPs	100/200/300	Lymphoma/lung cancer	*In vivo*
[56]	T cell	Injecting and hitchhiking T cell *in vivo*	Curcumin/aPD1/PEG NPs	43-50	Melanoma	*In vivo*
[65]	T cell	Encaps.	AuNPs	45	Lymphoma	*In vivo*
[70]	T cell	Encaps.	Dox/TargetMAG NPs	50	N/A	*In vitro*
[17]	NK	BP	PTX/liposome NPs	220	Ovarian cancer	*In vivo*
[42]	NK	BP	TRAIL/anti-CD57/liposome NPs	161	Prostate/breast/colon cancer	*In vitro*
[57]	NK	Injecting and hitchhiking NK *in vivo*	Trail/anti-NK1.1/liposome NPs	138	Melanoma, colon cancer	*In vivo*
[18]	MA	Encaps.	Dox/SiO_2_ NPs	28.4	Glioblastoma	*In vivo*
[25]	MA	Encaps.	Au/BSA nanorods	7	Liver cancer	*In vivo*
[30]	MA	Encaps.	Dox/liposome NPs	150	Lung cancer	*In vivo*
[47]	MA	BP	Fluorophores	N/A	Breast cancer	*In vivo*
[64]	MA	Encaps.	Dox/PLGA NPs	141.6	Glioblastoma	*In vivo*
[67]	MA	Encaps.	AuNRs & Dox/liposome NPs	145	Breast cancer	*In vivo*
[68]	MA	Encaps.	Dox only	N/A	Breast cancer	*In vivo*
[71]	MA	Encaps.	PTX/Fe_3_O_4_/liposome NPs	110.36	Breast/colon cancer	*In vitro*
[73]	MA	Encaps.	SN-38 NPs	119.13	Lung/breast cancer	*In vivo*
[44]	MO	Encaps.	Polystyrene microbeads	100/300/1000	N/A	*In vitro*
[45]	MO	Encaps.	RGD/cy5.5/PEG-SWNT	0.8-1.2	Glioblastoma	*In vivo*
[49]	MO	BP	LbL disk (500 nm thick)	7000	Inflamed lung	*In vivo*
[72]	MO	Encaps.	Dox/poly(AAc-co-DSA) NPs	200-260	Prostate cancer	*In vivo*
[6]	NSC	BP	Docetaxel/PEG-PDPAEMA NPs	400	Breast cancer	*In vivo*
[19]	MSC	Bioengineered	Fluorescence	N/A	Liver/lung cancer	*In vivo*
[40]	MSC	Encaps.	Quantum dots/PEG NPs	14.5	Breast cancer	*In vivo*
[41]	MSC	Bioengineered	IFN-*α*	N/A	Melanoma	*In vivo*
[52]	MSC	BP	Dox/silica nanorattle	152.9	Glioblastoma	*In vitro*
[53]	MSC	BP	Curcumin/chitosan NPs	377	Lung cancer	*In vivo*
[58]	MSC	BP	FluoSpheres	40	Liver cancer	*In vitro*
[69]	MSC	Encaps.	PTX/PLGA NPs	135.3	Glioblastoma	*In vivo*
[74]	MSC	Encaps.	PTX/PLGA/TAT NPs	225	Lung cancer	*In vivo*
[23]	RBC	Encaps.	ICG-BSA NPs & free Dox	N/A	Glioblastoma	*In vitro*
[24]	RBC	BP	Ferritin/ZnF16Pc NPs	15-18	Glioblastoma	*In vivo*
[46]	RBC	Both	Free Dox (in), Ce6 (on membrane)	N/A	Breast cancer	*In vitro*
[48]	RBC	Both	ICG/BSA (in), upconversion NPs (on membrane)	40	Liver cancer	*In vivo*
[61]	RBC	BP	PS or LDNG NPs	171/268	N/A	*In vitro*

Encaps. = encapsulation; BP = backpack. For other abbreviations, please refer to the abbreviation list.

**Table 4:** Different cell derivatives loaded with varied cargos for cancer diagnosis and therapy.

Refs.	Cell type	Loading method	Drugs/NPs	Drug/NP size (nm)	Cancer type	*In vivo*/*in vitro*
[32]	NK membrane	Coating	Gadolinium/PLGA NPs	109	Breast cancer	*In vivo*
[79]	MO membrane	Coating	Silicon particles	3200	Melanoma	*In vivo*
[80]	MA membrane	Coating	Dox/IND/Ce6/PEG/bilirubin complex	107	Breast cancer/melanoma	*In vivo*
[81]	MA membrane	Coating	PTX-albumin NPs	138.7	Melanoma	*In vivo*
[82]	MA membrane	Coating	Dexamethasone	N/A	Inflamed ear	*In vivo*
[83]	RBC membrane	Coating	Dox/Kirenol/phosphorous quantum dots	10	Cervical cancer	*In vivo*
[86]	Tumor cell membrane	Coating	AuNPs	40	N/A	*In vitro*
[22]	RBC sEVs	Encaps.	Free clodronate	N/A	CD47^−/−^model	*In vivo*
[95]	Blood sEVs	Between lipid layers	Free Dox	N/A	Liver cancer	*In vivo*
[96]	T cell sEVs	N/A	Chimeric antigen receptor	N/A	Breast cancer	*In vivo*
[101]	Tumor cell sEVs	Encaps.	ZnO nanocrystals	91	KB cancer	*In vitro*
[102]	Blood sEVs	Both	Dox/miRNA21 inhibitor (in), MTf/L17E (on EVs)	106	Glioblastoma	*In vivo*
[103]	RBC sEVs	Encaps.	RNA	N/A	Breast cancer	*In vivo*
[104]	Cancer sEVs	Encaps.	Free methotrexate	N/A	CCA	*In vivo*
[87]	Artificial RBC	Encaps.	Hemoglobin-dopamine complex	100	Breast cancer	*In vivo*

Encaps. = encapsulation; BP = backpack. For other abbreviations, please refer to the abbreviation list.

## Abbreviations

aPD1: Anti-PD-1 monoclonal antibody
ATP: Adenosine triphosphate
Au: Aurum
AuNR: Aurum nanorod
BBB: Blood-brain barrier
BSA: Bovine serum albumin
CARs: Chimeric antigen receptors
CCA: Cholangiocarcinoma
CCL-2: C-C motif chemokine ligand 2
CCL-5: C-C motif chemokine ligand 5
CCL-7: C-C motif chemokine ligand 7
CCL-8: C-C motif chemokine ligand 8
CCL-12: C-C motif chemokine ligand 12
CCL-25: C-C motif chemokine ligand 25
CCR7: C-C motif chemokine receptor 7
CD62L: L-selectin or lectin adhesion molecule 1
Ce6: Chlorin e6
CSF-1: Colony-stimulating factor 1
CXCL9: C-X-C motif chemokine ligand 9
CXCR4: C-X-C motif chemokine receptor 4
DDS: Drug delivery system
Dox: Doxorubicin
ECM: Extracellular matrix
ECs: Endothelial cells
EGF: Epidermal growth factor
EPR: Enhanced permeability and retention
EVs: Extracellular vesicles
FasL: Fas ligand
FDA: Food and Drug Administration
GDF-15: Growth differentiation factor
H: Hour
Her2: Human epidermal growth factor receptor 2
HGF: Hepatocyte growth factor
ICAM: Intercellular cell adhesion molecule
ICAM-1: Intercellular cell adhesion molecule 1
ICG: Indocyanine green
IFN-*γ*: Interferon *γ*
IL-1: Interleukin-1
IL-15Sa: Interleukin-15 superagonist
IL-17: Interleukin-17
IL-1*β*: Interleukin-1*β*
IL-2: Interleukin-2
IL-7: Interleukin-7
IL-8: Interleukin-8
IND: Indoleamine 2,3-dioxygenase 1 inhibitor
LDNG: Lysozyme-dextran nanogels
LFA-1: Lymphocyte function-associated antigen 1
LFA-1 (*α*L*β*2): Lymphocyte function-associated antigen 1, *α*L*β*2
M1: Macrophage phenotype 1
M2: Macrophage phenotype 2
Mac-1 (*α*M*β*2): Macrophage-1 antigen, *α*M*β*2
MAs: Macrophages
MOs: Monocytes
MSCs: Mesenchymal stem cells
MTD: Maximum tolerated dose
NEs: Neutrophils
NETs: Neutrophil extracellular traps
NIR: Near-infrared
NKG-2D: Natural killer group protein 2 family member D
NKp30: Natural killer cell p30-related protein
NKs: Natural killer cells
NPs: Nanoparticles
OVA-1: Ovalbumin-1
PBS: Phosphate-buffered saline
PD-1: Programmed cell death protein 1
PDGF: Platelet-derived growth factor
PDGF-*α*: Platelet-derived growth factor *α*
PDGF-*β*: Platelet-derived growth factor *β*
PD-L1: Programmed cell death ligand 1
PDT: Photodynamic therapy
PEG: Polyethylene glycol
PG: Polyglycerol
PLGA: Poly(lactic-co-glycolic acid)
PS: Polystyrene sphere
PSGL-1: P-selectin ligand 1
PTX: Paclitaxel
RBCs: Red blood cells
RES: Reticuloendothelial system
RGD: Arginine-glycine-aspartic
ROS: Reactive oxygen species
RT: Room temperature
siRNA: Small interfering RNA
SMAPs: Supramolecular attack particles
SN-38: 7-Ethyl-10-hydroxycamptothecin
SWNT: Single-walled nanotubes
TAT: Transactivator of transcription
TCRs: T cell receptors
TNF-*α*: Tumor necrosis factor *α*
TRAIL: Tumor necrosis factor-related apoptosis-inducing ligand
TSP1: Thrombospondin-1
VCAM: Vascular cell adhesion protein
VEGF: Vascular endothelial growth factor
WHO: World Health Organization.
